# Effect of Adipose-Derived Stem Cells and Their Exo as Adjunctive Therapy to Nonsurgical Periodontal Treatment: A Histologic and Histomorphometric Study in Rats

**DOI:** 10.3390/biom8040167

**Published:** 2018-12-10

**Authors:** Ebtehal Mohammed, Eman Khalil, Dina Sabry

**Affiliations:** 1 Lecturer of Oral Medicine, Oral diagnosis and Periodontology, Faculty of Dentistry, Beni Suef University, Beni Suef 62511, Egypt; 2 Lecturer of Oral Medicine, Oral diagnosis and Periodontology, Faculty of Dentistry, British University, Cairo 11837, Egypt; emankhalil@hotmail.co.uk or Eman.Khalil@bue.edu.eg; 3 Professor of Biochemistry, Faculty of Medicine, Cairo University, Cairo 11562, Egypt; dinnasabry69@yahoo.com or dinasabry@kasralainy.edu.eg

**Keywords:** nonsurgical periodontal treatment, adipose-derived stem cells, Exo., adjunctive periodontal therapy, rats, histologic study

## Abstract

Scaling and root planing (SRP) is of limited value in many cases, so adjunctive treatment was applied to augment its outcome. Adipose-derived stem/stromal cells (ADSCs) were investigated in periodontal regeneration with promising results. However, they have safety concerns. The exosomes (Exo.), which are extracellular vesicles mediating the action of stem/stromal cells, represent a new approach to overcome these concerns. Ligature-induced periodontitis was induced in 50 rats for 14 days, and they were divided into control (5 healthy rats for histologic comparison), SRP group, ADSCs group, and Exo. group, with evaluation intervals at 2 days, and 2 and 4 weeks, including 5 rats in each interval for each group. The specimens were evaluated for histologic description (H&E), histochemical study (Masson trichrome), and histomorphometric study, to evaluate the area % of newly formed tissues. The Exo. group revealed the best results in all intervals with significantly higher area % of newly formed tissues, followed by ADSCs and, finally, SRP. Both Exo. and ADSCs showed organized newly formed tissues with the Exo. group obtaining comparable histologic results to the normal, healthy tissues by 4 weeks. Adipose-derived stem/stromal cells and their Exo. represent a promising adjunctive treatment to SRP.

## 1. Introduction

Periodontitis is a chronic immune inflammatory disease of supporting tooth structures initiated by dysbiotic polymicrobial dental biofilm in a susceptible host [1]. The disease progression leads to attachment loss with the destruction of periodontal tissues and, finally, tooth loss [2]. Also, the periodontal diseases may impact many systemic conditions, including diabetes mellitus, cardiovascular disorders, and autoimmune diseases, e.g., rheumatoid arthritis [3].

Regeneration is defined as the reproduction or reconstitution of a lost or injured part of the body, in such a way that the architecture and function of the lost or injured tissues are completely restored. However, few techniques can be regarded as regenerative methods in periodontics, including biologics [4]. To achieve periodontal regeneration, a complex process of migration, proliferation, and function of different cells, in coordinated manner, should be enhanced [5].

The nonsurgical periodontal treatment includes scaling and root planing (SRP) as a basic procedure, which aimed at mechanical removal of the dental biofilm. However, it is of limited effect in the deeper periodontal pockets and inaccessible areas, where extra surgical interventions are indicated [6]. The adjunctive treatment depends mainly on antimicrobial mechanisms to augment the SRP results [7].

A tissue engineering approach for tissue regeneration implements four elements, including blood supply, progenitor cells, proper signaling molecules, and suitable scaffold [8]. Among the stem/stromal cells, the adipose-derived stem/stromal cells (ADSCs) represent a very attractive source for regenerative medicine, wherein they can be harvested in a massive amount with minimal invasiveness with no ethical concern, could differentiate into different cell types, and have immunemodulatory, protective, and antimicrobial effects, as reviewed by Kocan B et al. [9]. All these actions are mediated by a superior secretome profile of cytokines and growth factors, and they had been investigated in the periodontal treatment with promising results, as reviewed by Trofin E, et al. [10] and Tassi SA et al. [11].

In attempts to overcome the safety considerations associated with biomaterials and cell-based therapy, exosomes (Exo.) have emerged as a cell-free therapeutic approach, which is suggested to be more safe as they are endogenous in origin [12]. They are lipid membrane-associated extracellular vesicles of 40–150 nm, and a density of 1.09–1.18 g/mL, and they are secreted by many cell types, including mesenchymal stem/stromal cells (MSCs), where they have a massive amount of Exo. to which the therapeutic effects of MSCs might be attributed. The suggested main mechanism of Exo. is mediated by internalization of them into the targeted cells, where they have the same therapeutic effects as MSCs, including trophic activity, angiogenic effect, antiapoptic effect, immunemodulatory, and antimicrobial effects [13]. They had been investigated in preclinical models, including skin wound healing, cardiovascular, liver, kidney disease, bone regeneration, and diabetes mellitus. Moreover, they have been investigated in human clinical trials with promising results [14]. To the best of our knowledge, no previous study has investigated either the therapeutic effect of Exo. in periodontal regeneration, or the effect of ADSCs on nonsurgical periodontal treatment. 

The aim of the current study was to investigate the therapeutic potential of both ADSCs and their Exo. to SRP in nonsurgical periodontal treatment as an adjunctive therapy. 

## 2. Materials and Methods

### 2.1. Experimental Animals

The study was conducted in theanimal house, Kasr Alainy, Cairo University, in accordance with the ethical guidelines Ethical approval number: CU/III/73/18]. The study included 50 adult male Abino Wistar rats, as referred to in Du J. et al. [15], weighing between 210 and 250 g, and their age ranged from 6 to 9 months. Each 5 rats were housed together in a wiring cage under standard conditions, during the experimental period, at room temperature (21 ± 1 °C) and humidity (50–55%), 12 h dark/light cycle, and they were fed the standard rat chow pellets, and water was available ad libitum. Moreover, the animals were observed daily for ligature placement.

### 2.2. Induction of Periodontitis

Periodontitis was induced in all rats in accordance with Ionel A. et al. [16], as the rats were anesthetized with ketamine hydrochloride (70 mg/kg) and xylazine hydrochloride (10 mg/kg), intraperitoneally. The 4/0 nonresorbable sterile silk threads were used to create a figure of eight ligature around the lower incisors for 14 days (Figure 1), to facilitate the biofilm retention and food accumulation, in order to induce periodontal disease around the lower incisors.

### 2.3. Adipose-Derived Stem/Stromal Cells and Their Exo. Preparation

Fat tissue was obtained through subcutaneous incision from both the omentum and the inguinal fat pad. The procedures of ADSCs and their Exo. preparation had been carried out in the Molecular Biology and Tissue Engineering Unit, Department of Medical Biochemistry, Cairo University, School of Medicine.

The excised fat tissue was hydrolyzed using collagenase type II (Sigma, St. Louis, MI, USA) dissolved in phosphate-buffered saline (PBS; Gibco/Invitrogen, Grand Island, NY, USA) at 37 °C for 2 h. Strainers, 2 µm, were used to remove any tissue debris, followed by centrifugation at 1000 rpm for 5 min to form a cell pellet which was cultured with Roswell Park Memorial Institute RPMI medium (Gibco BRL, Waltham, MA, USA), 10% fetal bovine serum (FBS, Gibco BRL, Waltham, MA, USA), and humidified in a cell culture incubator containing 5% CO_2_ at 37 °C. Then, at 80–90% ADSC confluence, they were detached with 0.25% trypsin-ethylenediaminetetraacetic acid (EDTA, Gibco BRL, Waltham, MA, USA), and resuspended in other flasks. At fourth passage, ADSCs were used in all experiments. The surface marker expression of adipose MSCs had been characterized, in culture, by their morphological spindle shape-like cells. Furthermore, they had been identified by flow cytometry (Beckman Coulter, CA, USA), in the fourth passage, to assess positivity of expression of CD29, CD90, and CD105, and lack of, or negativity for, CD45 expression. To this end, they were trypsinized and adjusted to 1 × 10^6^ cells/mL cells, followed by incubation with 10 μL of monoclonal antibodies: CD45 fluorescein isothiocyanate FITC, CD29 phycoerythrin PE, CD105 PE, and CD90 PE (Beckman Coulter, CA, USA) at 4 °C in the dark, and the same species isotypes served as a negative control ().

The Exo. had been obtained from the supernatants of the third passage ADSCs (5 × 10^6^ cells/mL) that were cultured in RPMI deprived of FBS and supplemented with 0.5% of bovine serum albumin (BSA) (Sigma). In order to remove the debris, the cell-free supernatant was first obtained by centrifugation at 2000× *g* for 20 min, then centrifuged at 100,000× *g* (Beckman Coulter Optima L 90K ultracentrifuge) for 1 h at 4 °C. Thereafter, the obtained pellet was washed in serum-free mediumcontaining HEPES 25 mM (Sigma), and submitted to a second ultracentrifugation under the same conditions. The quantification of protein content was done by the Bradford method (BioRad, Hercules, CA, USA). After that, the purified extracellular vesicles (EVs) were cultured overnight in the medium used for collection of EVs. Electron microscope analysis was done, where the images were obtained at a working distance of 15 to 25 mm, and an accelerating voltage of 20 and 30 kV, where the digital acquisition and analysis were performed using the JEOL T300 system (Musashino, Akishima, Tokyo). Flow cytometry analysis was performed using the following FITC-conjugated antibodies: CD83 (Miltenyi Biotec, Bergisch, Germany) and CD73 (Becton Dickinson, NJ, USA), and FITC mouse non-immune isotypic IgG (Dako Cytomation, Glostrup, Denmark) was used as a control [17].

### 2.4. Study Groups

After 14 days, the experimental animals were randomly assigned to one of the following four groups:

Control group: 5 normal healthy rats, without any intervention for the descriptive study (H&E stain); accordingly, they were not included in histochemical and histomorphometric studies.

Scaling and root planing (SRP) group: 15 rats that had received scaling and root planing only.

ADSC group: 15 rats that had received scaling and root planing and ADSCs (1 × 10^7^) suspended in 200 µL PBS (phosphate-buffered saline), and injected locally into the pocket using a disposable plastic syringe, as an adjunctive treatment.

Exo. group: 15 rats had received scaling and root planing and ADSC exosomes (80–150 µg protein suspended in 200 µL PBS), injected locally into pockets using a disposable plastic syringe, as an adjunctive treatment. 

The animals were allowed to heal for intervals of 2 days (5 animals per each group), 2 weeks (5 animals per each group), and 4 weeks (5 animals per each group), and then they were anesthetized and sacrificed by cervical dislocation. 

### 2.5. Histologic and Histochemical Preparation

After the sacrifice at the assigned dates, the samples were extracted from animals and were preserved in 10% formalin for 72 h. Then, they were decalcified using 20% formic acid for a period that ranged from 2 to 4 weeks. Thereafter, the decalcified samples were embedded in paraffin, where the serial sections, 5 mm thickness in the mesiodistal direction, were prepared and stained with hematoxylin and eosin (H&E) for descriptive analysis, and Masson’s trichrome for histochemical analysis, where the newly formed collagen and osteoid were represented with blue or green reaction, and cellular cytoplasm represented by red reaction.

### 2.6. Histomorphometric and Statistical Analysis

All the histochemically stained sections were examined by a light microscope, using an image analyzer computer system with software (Leica, Wetzlar, Germany), where the area containing the most uniform positive histochemically stained tissues were selected for evaluation of area %, using magnification 200× at five points, where one point in each slide for each group interval was selected. Then, they were calibrated automatically to convert the measurement units (pixels) produced by the image analyzing program into actual micrometer units, in order to be tabulated and statistically evaluated using one-way ANOVA test and the post hoc Tukey test, and the mean values of data ± standard deviation were expressed and a *p*-value was calculated to determine significance, which was done using statistical package for the social science SPSS computer system version 9. 

## 3. Results

### 3.1. Descriptive Histologic Results

The two day interval reflects the early healing events, including the inflammatory reaction, while the two and fourweek intervals reflect the healing represented in newly formed cementum, periodontal fibers, and alveolar bone. 

After the two day interval, all groups showed infiltration of inflammatory cells to different degrees, where there was a mixture of neutrophils and mononuclear cells (lymphocytes and macrophages). In the SRP group, there was abundant inflammatory infiltration in the periodontal tissues (Figure 2a), while the inflammatory infiltration in ADSC group was less than SPR group (Figure 2b). In Exo. group, the inflammatory infiltration was the least observed among all groups, and there were signs of periodontal tissue formation, which was a striking finding, represented by proliferating periodontal fibroblasts and the alveolar bone showing multiple reversal lines and newly formed osteoid tissue (Figure 2c,/C).

After the two week interval, all groups show formation of new periodontal tissues with different degrees of proliferation and organization. In the SRP group, there were multiple large blood vessels in periodontal space, with less evidence of proliferating periodontal cells, while the newly formed bone trabeculae were disorganized with a layer of osteoid tissue (Figure 3a). In the ADSC group, the periodontal tissue was highly cellular and disorganized, while the alveolar bone showed multiple reversal lines with narrow spaces and a thick layer of osteoid tissues (Figure 3b). The Exo. group showed the most evident proliferation in periodontal tissue, with increased cellularity and significant organization, also, the alveolar bone was more organized with an osteoid tissue layer (Figure 3c,/C).

After the four week interval, in comparison to normal, healthy periodontal tissue of control group (Figure 4a), the SRP group was the least organized one in healing (Figure 4b). The ADSCs showed highly cellular periodontal tissue, with the cells are perpendicular to the cementum and alveolar bone, and the most characteristic finding was multiple blood vessels formation (Figure 4c,/C), while the Exo group showed the most healing signs, represented in periodontal tissues with normal width, well-oriented periodontal cells and fibers (Figure 4d). 

### 3.2. Histochemical and Histomorphometric Results

The Exo. group revealed the most dense reaction, indicating formation of new collagen, osteoid, and cellular proliferation in an organized pattern during all three intervals, followed by ADSCs group, while the SRP group showed the weaker reaction among the study groups, and these results were represented statistically.

The ANOVA test showed significant difference between all groups, Table 1, while the post hoc Tukey test revealed that the area % of newly formed tissues in Exo. group was significantly higher than those of both ADSCs and SRP for all experimental intervals (2 days, 2 weeks, and 4 weeks). Also, ADSCs was significantly higher than SRP group, in all intervals. Table 2, Table 3 and Table 4, Figure 5. 

## 4. Discussion

This is the first study to investigate the therapeutic effect of Exo. in periodontal treatment, generally. Also, it is the first study to investigate the effect of ADSCs in nonsurgical periodontal treatment.

The animal study provides a valuable tool for examining the effect of new therapeutic regenerative techniques in periodontics, especially using small animals, with many advantages, including cost effectiveness and simplicity of handling [18], where the rat model provides an attractive model for these studies, due to the histological similarity of their periodontium to human, with the exception of keratinization of the gingival sulcus [19]. The rat incisor model provides many advantages over molars, including simplicity, accessibility to the daily observation of ligature integrity without trauma or need for general anesthesia, and reproducible disease induction within 14 days [16].

The inflammatory phase represents the early wound healing events during the first 3 days, and it functions mainly in wound debridement during the early phase and, additionally, in the late phase, the macrophages contribute to wound healing via release of various growth factors targeting the involved cells in the tissues’ formation as fibroblasts [20]. As both ADSCs [21] and their Exo. [22] have immunomodulatory effects with an anti-inflammatory effect, it was important to evaluate their effects on the inflammatory phase of healing. Moreover, by 14 days, all periodontal tissues had been formed, and they mature, with time, to reach the normal thickness and function after periodontal surgery in rats, so the 2 and 4 week intervals were selected to investigate the newly formed periodontal tissues [23].

The SRP represents the basic procedure in periodontal treatment by elimination of the bacterial biofilm, leading to decrease in the bacterial load and creation of a more favorable environment for periodontal healing [7]. However, it cannot be regarded as a regenerative technique, as the histologic studies showed that the healing after SRP by long junctional epithelium is mainly predictable, although there is some formation of new connective tissue attachment [24].

The ADSC group in the current study showed better results, with significantly higher area percentage of newly formed periodontal tissues than SPR, showing more proliferation and organization in all intervals. These results are similar to our previous study [25], and the results of other studies as reviewed by Bassir S. et al. [26] and Intini G. [26]. However, most of these studies investigated ADSCs in periodontal surgical animal models, where only a few studies investigated the effect of stem/stromal cells in nonsurgical treatment, such as the study by Lemaitre M. et al. [27], which showed newly formed periodontal tissues, except alveolar bone, that might be explained by the osteogenic potential of ADSCs that could be affected by many factors, including the source and method of extraction, culture, and in vivo microenviroment [9], and another study, by Du J. et al. [15], that investigated the effect of the allogenic bone marrow stem/stromal cells in nonsurgical models with evidence of anti-inflammatory and healing effects. The regenerative effects of ADSCs include cell engraftment effect by cell differentiation and proliferation. However, it represents a minor trophic effect, as they have superior secretion of a wide range of bioactive molecules, enhancing the endogenous regeneration by different cell types’ migration, differentiation, and proliferation, including fibroblasts, endothelial, and epithelial cells [28], a superior angiogenic effect to other mesenchymal stem/stromal cells [29] and, finally, they provide protective and supportive effects by reducing apoptosis, fibrosis, and inflammation [30].

The Exo. group of the current studies showed a striking result by evidence of new periodontal tissue formation in the 2 day interval, that was represented in proliferating primitive periodontal fibroblast and osteoid tissues while, on the other hand, there was minimal evidence of inflammatory cells, that can be explained by the anti-inflammatory effects of exosomes [22]. Also, the results of both 2 and 4 weeks were the best, as the area % of newly formed tissues were significantly higher than SRP and ADSC groups, with highly organized structures that were comparable to normal healthy tissues by 4 weeks. The effect of Exo. to shorten the rate and improve the quality of wound healing had been revealed by other studies on skin wound healing applying ADSC Exo. [31] and umbilical cord stem cells [32]. They explained these results by the ability of Exo. to be taken by the targeted cells in a dose-dependent manner, enhancing the migration, proliferation, and function of fibroblasts and endothelial angiogenesis. Consistent with Vizoso et al. [13], the Exo. provide many advantages over stem/stromal cell therapy, through being biologics that are ready to be used, having extra shelf life in storage, being more safe as they are endogenous molecules, whilst the cell therapy by transplantation of living and proliferative cells have many potential risks, consisting of tumorigenicity, immune compatibility and, moreover, they can be prepared in laboratories from cell culture under strict conditions to be more economical, safer, and ready for use in acute conditions.

## 5. Conclusions

In the current study, both ADSCs and Exo. represent promising regenerative techniques that can be used as an adjunctive treatment to SRP, enhancing the outcome of the nonsurgical periodontal treatment. Exo. showed superior results to ADSCs, with the additional advantages of safety and easy preparation. They can be applied as a suspension injected locally to periodontal defects, without the need or additional cost of preparation of a scaffold.

## Figures and Tables

**Figure 1:** This figure shows the figure eight ligature around the lower incisors.

**Figure 2:** Two days interval. (**a**) Photomicrograph of the scaling and root planing (SRP) group showing numerous inflammatory cells infiltrating the periodontal ligament and disorganized bone trabeculae (H&E 400×); (**b**) Photomicrograph of the adipose-derived stem/stromal cell (ADSC) group showing numerous inflammatory cells infiltrating the periodontal tissues (yellow arrow) (H&E 400×); (**c**) Photomicrograph of the exosomes (Exo.) group showing a large periodontal ligament space filled with a disorganized proliferating periodontal ligament tissue (H&E 400×) and attached to a regular cementum surface. Osteoid tissue (blue arrows) is formed on the bone surface (H&E 400×) in (**/C**).

**Figure 3:** Two week interval. (**a**) Photomicrograph of SRP group showing dilated blood vessels in the periodontal ligament (red arrow) attached to a regular cementum layer, and an irregular bone surface with a layer of osteoid (yellow arrow) (H&E 400×); (**b**) Photomicrograph of ADSC group showing irregularly proliferating periodontal tissue, attached to a regular surface of cementum, and disorganized bone trabeculae showing few cells and many reversal lines (blue arrow) (H&E 400×); (**c**) Photomicrograph of Exo. group shows the interdental periodontal ligament space filled with an organized proliferating periodontal ligament tissue (yellow arrow) (H&E 200×); (**/C**) Photomicrograph showing a periodontal ligament with an organized proliferating periodontal ligament tissue attached to a regular cementum surface with formation of osteoid tissue (blue arrow) (H&E 400×).

**Figure 4:** Four weeks interval. (**a**) Control group: Photomicrograph showing the normal periodontal healthy tissues (H&E 200×); (**b**) Photomicrograph of SRP group showing healed periodontal ligament tissue with wide periodontal space and periodontal cells which are lower in number and not organized (H&E 400×); (**c**) Photomicrograph of ADSCs group showing highly well-organized proliferating periodontal tissue perpendicular to the cementum and bone (yellow arrows) (H&E 400×), multiple blood vessels (white arrow) and osteoid tissue, as shown in (**/C**); (**d**) Photomicrograph of Exo. group shows a narrow periodontal ligament space of uniform thickness filled with a highly organized proliferating periodontal ligament tissue attached to a regular cementum surface and well-formed dense healthy bone (H&E 400×).

**Figure 5:** Bar chart showing area percent values of the studied groups after different time intervals.

**Table 1:** Comparison of mean area % values of newly formed tissues for the studied groups (ANOVA test).

	SRP Group	ADSC Group	Exo. Group	*p-*Value
2 days	7.29 ± 1.34	13.1 ± 2.81	21.9 ± 1.97	*p* = 0.001 *
2 weeks	11.6 ± 1.14	18.2 ± 1.38	26.8 ± 2.12	*p* = 0.001 *
4 weeks	13.4 ± 2.30	23.0 ± 2.85	32.1 ± 3.5	*p* = 0.001 *

* Significance is set at *p* < 0.05

**Table 2:** Pairwise comparison of mean area % values of newly formed tissues for the studied groups after 2 days (post hoc Tukey test).

Groups	SRP Group	ADSC Group	Exo. Group
SRP group	−	*p* = 0.0001 *	*p* = 0.0005 *
ADSC group	*p* = 0.0001 *	−	*p* = 0.0001 *
Exo. group	*p* = 0.0005 *	*p* = 0.0001 *	−

* Significance is set at *p* < 0.05.

**Table 3:** Pairwise comparison of mean area % values of newly formed tissues for the studied groups after 2 weeks (post hoc Tukey test).

Groups	SRP Group	ADSC Group	Exo. Group
SRP group	−	*p* = 0.0001 *	*p* = 0.0001 *
ADSC group	*p* = 0.0001 *	−	*p* = 0.0001 *
Exo. group	*p* = 0.0001 *	*p* = 0.0001 *	−

* Significance is set at *p* < 0.05.

**Table 4:** Pairwise comparison of mean area % values of newly formed tissues for the studied groups after 4 weeks (post hoc Tukey test).

Groups	SRP Group	ADSC Group	Exo. Group
SRP group	−	*p* = 0.0006 *	*p* = 0.0001 *
ADSC group	*p* = 0.0006 *	−	*p* = 0.0010 *
Exo. group	*p* = 0.0001 *	*p* = 0.0010 *	−

* Significance is set at *p* < 0.05.
